# Particle Swarm Algorithm and Its Application in Tourism Route Design and Optimization

**DOI:** 10.1155/2022/6467086

**Published:** 2022-03-29

**Authors:** Bing Lu, Chunlei Zhou

**Affiliations:** ^1^Tourism Management, Zhengzhou Tourism College, Zhengzhou 450000, China; ^2^Henan Polytechnic, Zhengzhou 450000, China

## Abstract

Most of the traditional tourism route planning algorithms only consider single-factor planning, that is, the influence of scenic spots on route planning. Particle swarm optimization algorithm is favored by many people because of its simple concept, easy implementation, and good robustness. Aiming at this problem, this paper takes the actual geographic data as the research object of the tourism route problem and describes the model of the discrete particle swarm algorithm based on geographic coordinates to solve the tourism route problem, which is used to solve practical problems. In order to further improve the global search ability of the algorithm, a self-balancing mechanism is proposed, which makes the algorithm process simple and the algorithm performance improved. At the same time, multithread parallelism is adopted to improve the solution speed of the algorithm, which makes up for the deficiency of the parallelization research of the algorithm.

## 1. Introduction

With the development of network technology, people now collect information on major tourism websites before traveling, but they can only obtain static locations and attribute information of scenic spots and hotels. Based on this information, designing a path plan that meets their own travel needs will cost a lot of money, time, and energy. Although a small number of travel websites also provide similar route planning functions, after selecting this function, most travel agency travel route product recommendations rather than regional travel route planning appear. Therefore, the public urgently needs a tourism route planning method that considers attractions, hotels, and other factors to meet the personalized and practical needs of tourists [1–6].

The path optimization ultimately needs to obtain a path that satisfies the optimization index, and the smoothness of the curve must be satisfied in any path planning problem. In order to generate a smooth and continuous curve, the Bezier curve, Ferguson curve, and 3 curve were used in the previous work to describe the path, the results were compared, and it was concluded that the algorithm of this subject (particle swarm optimization algorithm) is more suitable for describing the path. *Curve*. The Bezier curve stands out because it is easy to satisfy the smoothness, and it is easier to change the direction when describing the path (that is, the curve is more flexible). Therefore, in the later work, the Bezier curve is used to describe the path, the path planning problem is transformed into the problem of optimizing the position of a finite number of points on the Bezier curve, and the optimal path search is performed through an improved particle swarm optimization algorithm.

In recent years, many scholars have conducted a lot of in-depth research on tourism route planning algorithms. Luo et al. [7] used the improved Dijkstra algorithm to realize the travel route planning. Some scholars transformed the travel route planning problem into a traveling salesman problem and used an improved ant colony algorithm to solve it, while others improved the ant colony algorithm [8–12].

With the development of artificial intelligence, the concept of swarm intelligence is introduced into optimization algorithms, which in turn promotes the emergence of intelligent algorithms such as particle swarm optimization algorithms. The easy calculation, fast convergence speed, strong global search ability, etc., have achieved good results in many multidimensional continuous space optimization problems. In order to apply to complex situations, the researchers improved the PSO and proposed two stages of PSO. The two paragraphs of PSO used in the literature are to expand the search domain and use the collaborative search of another group composed of multiple subgroups and the optimal solution in each subgroup, thereby improving the algorithm's global search capability. There are also two paragraphs of PSO in the literature that optimize different objective functions in two different stages. In addition, the path obtained in the literature is formed by connecting multiple Ferguson splines and only realizes C1 continuity; that is, the acceleration magnitude at the connection will change suddenly, and there will be an unreal feeling in the virtual scene [13–18]. At present, the solution process of the PSO algorithm used to solve the TSP problem is relatively complex and the solution speed is slow. The experimental results cannot explain the advantages of the overall performance of the algorithm, and the experiments are mostly based on test data. Therefore, some people take the actual geographic data as the research object of the TSP problem and describe in detail the model of the discrete PSO algorithm based on geographic coordinates to solve the TSP problem, which is used to solve practical problems. In order to further improve the global search ability of the algorithm, a self-balancing mechanism is proposed, which makes the algorithm process simple and the algorithm performance improved. At the same time, multithread parallelism is adopted to improve the solution speed of the algorithm, which makes up for the deficiency of the parallelization research of the algorithm.

The particle swarm algorithm has been used to solve many optimization problems. The original or standard particle swarm algorithm is mainly suitable for solving the optimization problem of the continuous solution space. However, with the emergence of actual requirements, the PSO algorithm has gradually been applied to the space of discrete solutions for different application fields. However, how to better apply the algorithm to the optimization problem of discrete space will be a difficult problem for particle swarm optimization [19–22]. Therefore, its development direction can be divided into the following categories:

1. Theoretical research on the PSO algorithm; the algorithm still lacks clear mathematical proofs. Using mathematical tools to analyze the algorithm will help the development of the theoretical foundation.
2. The application of the PSO algorithm in new fields, according to the variability of actual problems, is not universal to solve practical problems and can only be determined by the user's experience.
3. The PSO algorithm solves actual problems based on actual data; at present, most of the related improvements of the algorithm are aimed at the algorithm rather than the specific actual problem. The algorithm should be developed for the specific problem instead of blindly solving it through the test data.

It can be seen that the existing tourism route planning research results are relatively large, but there are still shortcomings. (1) The limiting factors are relatively fixed, and the impact of multiple practical factors is not considered. For example, most algorithms only plan tourism routes based on scenic spots, and the actual travel process did not consider the impact of the important factor “hotel”, which caused the applicability of the route planning results to decline. (2) Most of the data in the algorithm is based on historical data, which does not fully take into account the individual needs of tourists. According to tourists' preferences and consumption levels, a personalized travel route planning program is generated [23, 24].

## 2. Particle Swarm Algorithm

The tourism route design is shown in Figure 1. At the IEEE Congress on Evolutionary Computation, particle swarm algorithm is on par with evolutionary algorithms such as genetic algorithm and evolutionary programming, and it exists as an independent branch. The earliest particle swarm optimization algorithm has a fast convergence speed, but it is easy to converge to a local optimum. In response to this shortcoming, many interesting and improved particle swarm optimization algorithms have been proposed. The main improvements are in the following three directions. One is to study and adjust the original particles or the update formula of the group optimization algorithm. The second is to change the topological structure between the constructed particles. The particle information or partial particle information is shown in Figure 2. The third is to construct a hybrid particle swarm optimization algorithm through the effective combination of other evolutionary algorithms and nonevolutionary algorithms.

With the continuous improvement of algorithm improvement, many experts and scholars are committed to applying the algorithm to practical optimization problems. In the past ten years, particle swarm optimization has been widely used in various optimization problems due to its superiority. In recent years, domestic research on particle swarm optimization algorithms has also achieved rapid progress, and the number of papers has increased significantly. Many scholars have tried to combine particle swarm optimization with other algorithms and have achieved good results in some application areas of social economy, science, and engineering. Effects, such as robot path planning, optimization of antenna parameter settings, enhancement of the contrast of gray images, fuzzy recognition of nonlinear system motion, training of neural networks, optimization of power distribution systems, and rearrangement of train numbers during traffic jams are difficult to describe. At the same time, many scholars are committed to applying particle swarm algorithms to hardware implementation.

However, traditional particle swarm optimization algorithms have shortcomings such as easy convergence to local optimal and premature. Therefore, in recent years, many improved algorithms have been proposed to overcome this shortcoming, such as adaptive weight PSO in UAV path planning the application of interval multiobjective PSO in path optimization, the application of PSO based on quantum genetic algorithm in diving path optimization, and the application of PSO with proportional integral derivative in robot path planning. These improved algorithms are all because their own characteristics are applied. Dynamic multigroup particle swarm optimization algorithm is widely used because its dynamic neighborhood structure overcomes the shortcomings of traditional PSO. Therefore, this topic uses a dynamic multigroup particle swarm optimization algorithm to solve the path optimization problem.

The vector and the position and velocity are, respectively, represented as

(1) $$\begin{array}{c} X_{i}={\left(x_{i}^{1},x_{i}^{2},x_{i}^{3},\ldots ,x_{i}^{n}\right)}^{D},\\ V_{i}={\left(v_{i}^{1},v_{i}^{2},v_{i}^{3},\ldots ,v_{i}^{n}\right)}^{D}, \end{array}$$

where *x* is the position and *v* is the speed. Then, the speed and position update equation is

(2) $$\begin{array}{c} \left\{\begin{array}{c} x_{i\;d}^{k+1}=x_{i\;d}^{k}+v_{i\;d}^{k+1},\\ v_{i\;d}^{k+1}=v_{i\;d}^{k}+c_{1}\mathrm{ran}d_{1}^{k}\left(p_{i\;d}^{k}-x_{i\;d}^{k}\right)+c_{2}\mathrm{ran}d_{2}^{k}\left(g_{i\;d}^{k}-x_{i\;d}^{k}\right), \end{array}\right. \end{array}$$

where *k* is the number of particle iterations; *v* is the velocity of the particle. Generally, in order to prevent the particle from moving away from the search space, the particle velocity range is specified; cl, *c*2, rand1, and rand2 are the random variables of the particle, which are called here. To learn the factor, the value can be an integer or an interval value, which represents the probability of a certain value of the particle; *x* is the position of the particle at the kth iteration; *p* is the individual optimal position of the particle itself; *g* is the particle the best overall position of the group.

The basic process of the original particle swarm is as follows:

1. *Initialization*. Initialize particle-related parameters, such as random variables, number of particles, particle position, and velocity. The setting of each particle is the current position, the fitness value of the particle is recorded, and the optimal fitness value of the particle swarm is recorded.
2. *Evaluation of Particles*. If the current individual fitness value of the particle is not as good as the evaluation value, update the individual extreme value and set the value to the particle position; if the current global extremum is not as good as the best of the individual optimal values of all particles, update the global extremum and set the value to the position of the particle group.
3. *Update Particles*. The velocity and position of the particles are updated by formula (2).
4. *End Optimization*. If the current number of iterations reaches the specified value, stop the iteration and output the most

excellent solution; otherwise, go to (2).

Subsequently, Kelmedy and Ebethart proposed a basic particle swarm optimization algorithm [25]. In the original particle swarm algorithm update formula model, a variable *w*, which is the inertia weight value, was added. This inertial weight value is used to balance the particle searchability. The particle update formula is very similar to formula (2), except that the inertia weight value is added to the velocity update formula. The particle adjusts its position according to

(3) $$\begin{array}{c} \left\{\begin{array}{c} x_{i\;d}^{k+1}=x_{i\;d}^{k}+v_{i\;d}^{k+1},\\ v_{i\;d}^{k+1}=wv_{i\;d}^{k}+c_{1}\mathrm{ran}d_{1}^{k}\left(p_{i\;d}^{k}-x_{i\;d}^{k}\right)+c_{2}\mathrm{ran}d_{2}^{k}\left(g_{i\;d}^{k}-x_{i\;d}^{k}\right), \end{array}\right. \end{array}$$

where the meaning of each variable is the same as that of formula (2). The first part of the velocity formula is the particle's previous speed, and the inertia weight value determines the retention of the particle's own speed; the second part is the particle's self-cognition process, which can retain its current optimal value; the third part is the particle group recognition. Knowing the process, the particles cooperate with each other to make the entire group achieve the optimal value. If the second part of the model is removed, then the entire particle will converge too fast at this time and easily fall into the local optimum; if the third part is removed, the entire particle does not have the ability of group cognition, and the probability of obtaining the optimal solution is very small. The end condition of the algorithm is generally selected as the maximum number of iterations or the optimal solution searched so far has met the predetermined minimum evaluation value, which is the fitness value.

The algorithm steps in the search and solution of the problem are also five steps, except that the inertia weight value is added to the particle update formula.

**Step 1 .**

Initialize the population size, search dimension, iteration times, inertia factor, learning factor, convergence accuracy, particle velocity range, and other parameters of the PSO algorithm according to the optimization problem.

**Step 2 .**

Randomly assign the position and velocity of each particle in the optimization space, and make the individual optimal position value of each particle default at the moment to the position value of the current particle.

**Step 3 .**

Use the fitness evaluation function of the optimization problem to calculate the fitness value of each particle for each generation. If the fitness value of the particle is better than the current individual extreme value of the particle, update the individual optimal position of the particle, and use the current particle's position. The particle's position value replaces the individual optimal position value. If the best value among the individual extreme values of all particles in the whole group is better than the current global optimum value, then let the global optimum position value replace the individual optimum position value, so as to complete the update of the global optimum value.

**Step 4 .**

Update the position and velocity of each particle in the PSO algorithm according to the formula, and reassign the particles that are out of bounds.

**Step 5 .**

Check whether the end condition is met. If the number of iterations at the moment reaches the upper limit, or the result of the optimization meets the accuracy required for convergence, and stop the iteration and output the optimal result; otherwise, the algorithm jumps to Step 3. When the particles generate the next generation. The update formula used is (3). Since the basic particle swarm algorithm was proposed, the updated formula model of the basic particle swarm algorithm has become the beginning of the improvement of the particle swarm algorithm, and many improvement strategies are developed based on this model. Because the essence of the particle swarm algorithm cannot be changed, it has its own characteristics.

The convergence of the particle swarm algorithm means that the algorithm approaches the end state, and the change of particle position becomes smaller with the increase of time and the change of speed in terms of the following form:

(4) $$\begin{array}{c} \underset{k⟶+\infty }{\lim}a_{k}=x^{*}. \end{array}$$

For example, the PSO algorithm can successfully find the local minimum in the area, which satisfies the following formula:

(5) $$\begin{array}{c} \underset{k⟶+\infty }{\lim}a_{k}=x_{D}^{*}. \end{array}$$

That is, the global optimal value found in the search process forms a sequence, and the sequence is convergent and converges to the above formula. This value belongs to the search space, but it does not indicate whether it is global or local. It is a necessary condition for the algorithm to end in the specified number of iterations, not a sufficient condition for convergence. How to analyze whether the algorithm meets the requirements of formula (4). The following will analyze the convergence of the particle swarm algorithm.

Taking the most commonly used update formula model of the PSO algorithm with inertia weight as an example, a series of analyses of its convergence will be carried out. The formula is as follows:

(6) $$\begin{array}{c} \left\{\begin{array}{c} x_{i\;d}\left(k+1\right)=x_{i\;d}\left(k\right)+v_{i\;d}\left(k+1\right),\\ v_{i\;d}\left(k+1\right)=wv_{i\;d}\left(k\right)+c_{1}\mathrm{ran}d_{i\;d}\left(k\right)\left(p_{i\;d}\left(k\right)-x_{i\;d}\left(k\right)\right)+c_{2}\mathrm{ran}d_{2}^{k}\left(g_{i\;d}\left(k\right)-x_{i\;d}\left(k\right)\right). \end{array}\right. \end{array}$$

This updated formula is mostly used for multiple particles, where *k* is generally defined as the number of iterations, that is, the number of updates, the subscript *i* represents the particle number, and *d* represents the dimension. In order to simplify the formula, both *i* and *d* are omitted. After simplification, the whereabouts of each individual particle can be analyzed, and the whole can be seen through the individual to analyze whether the particle is convergent. Substituting the first formula in formula (6) into the second formula gives the following formula:

(7) $$\begin{array}{c} x_{k+1}=x_{k}+wv_{k}+\phi_{1}\left(p_{k}+x_{k}\right)+\phi_{2}\left(g_{k}+x_{k}\right), \end{array}$$

where

(8) $$\begin{array}{c} \phi_{1}=r_{1}\left(k\right)c_{1},\phi_{2}=r_{2}\left(k\right)c_{2}. \end{array}$$

Then,

(9) $$\begin{array}{c} x_{k+1}=\left(1-\phi_{1}-\phi_{2}\right)x_{k}+\phi_{1}p_{k}+\phi_{2}g_{k}+wv_{k}. \end{array}$$

Obtained by formula (6), we can get

(10) $$\begin{array}{c} v_{k}=x_{k}-x_{k-1}. \end{array}$$

Substituting it into (9), we can get

(11) $$\begin{array}{c} x_{k+1}=\left(1+w-\phi_{1}-\phi_{2}\right)x_{k}+\phi_{1}p_{k}+\phi_{2}g_{k}-wv_{k-1}. \end{array}$$

The common particle swarm algorithm improvements are based on inertia weight value improvement, based on learning factor improvement, based on genetic thinking, and based on ant colony algorithm thinking. In the improvement of the particle swarm algorithm based on the inertial weight value, according to formula (3), the first part of the first formula shows that the particle has the ability to retain its own flight speed and is affected by the influence of *w* inertia weight value. At present, there are three methods to modify the inertia weight value: linear decrement method, fuzzy method, and random method. The linear decrement method works well when testing the unimodal function, but when the function is multipeak, the effect is not good; the fuzzy method is better than the linear decrement method when optimizing the unimodal function, but the effect is still not good when the multipeak function is optimized. Good, it is difficult to find a good inertial weight value; the random method is relatively simple, and it can find a good solution in many function optimizations and is used by many applications.

In the algorithm improvement based on learning factors, the learning factors c1 and c2 increase the particle convergence speed, but they are also prone to fall into local optimal values when optimizing multipeak functions. Therefore, in order to balance the local searchability and the global search ability, in general, cl = c2, or in special problems, cl and c2 belong to the interval [0, 4]. In the improvement of the algorithm based on genetic ideas, Wang and Fan [1] proposed a cross-particle swarm algorithm. In the standard particle swarm update formula, parameters were added to reduce the number of speed updates. In order to avoid premature phenomena, the algorithm also eliminated some values and changed convergence speed. However, this method only increases the complexity of the algorithm and does not take discreteness into consideration. In the improvement based on the idea of ant colony algorithm, Beed et al. [26] proposed a hybrid ant colony particle swarm optimization algorithm and applied it to solve flexible job shop scheduling problems, and his analysis and experiments confirmed the convergence of this algorithm. Therefore, no matter what the problem is, the algorithm must be modified for the specific problem to get the desired result.

## 3. System Design and Implementation

This method of solving problems for specific data has verified its feasibility and effectiveness through experiments and provides some ideas for parallel processing of problems, instead of blindly improving through parallel tools like most current parallel models. The performance of the computer ignores the actual problem to be solved. At present, the method of solving path problems through the PSO algorithm has been initially developed, and some new ideas have been proposed for the improvement of the PSO algorithm, but in the end, the path problems solved by these algorithms are seldom tested through actual data, and most of them use them. What is the test data; these test data have basically met the sufficient conditions required to solve the problem. In the face of actual data, these improved PSO algorithms are basically helpless, because their initial focus is not actual specific problems, but PSO algorithms. Their design thinking is a process from algorithm to problem, unlike the design thinking of this article, which is a process from problem to algorithm and then to problem. Coupled with the parallelization of the algorithm when solving the path problem in this article, it is to improve the speed of solving the problem by using parallel tools for specific problems. There has been considerable progress in parallel processing. High-performance computing and clusters have also appeared hybrid parallel models such as MPL and OPE. However, the main focus of these parallel environments and models is the computer. What is the problem? Improve computer performance. The experimental verification of these models is mostly based on the hardware aspects such as chips or some mathematical test functions such as Jacobi iteration by some large companies. Large-scale projects generally use 8 or 16 multimachine clusters, and the test functions generally use 4 nodes and 2 node's multicore computer. No matter which method is adopted, the focus of these parallel models is mainly on the computer, and there is no parallel model for the actual problem solved in this paper. The application system model here is designed in this paper for the actual data and PSO algorithm to solve the TSP problem, including the algorithm parameter setting area and the TSP problem application area, there is parallel processing in the application area, and the computer is effectively improved through this parallelism. The rate of solving specific application problems improves the accuracy of the solution results and the rate of problem solving. The predicted value is shown in Figure 3.

In order to effectively reflect the solution results of the problem in the system and will not interfere with each other, the system is mainly composed of three parts, including data area, parameter area, and TSP problem area. The data in the data area consists of 3 map layers: Wuhan city tourist attractions data, Wuhan city road network data, Wuhan city building area. The data display is loaded into the application system through the map operation software. After the data is loaded, the basic operations on the data can be performed on the system through the map operation software: zoom in, zoom out, move, and load. The parameter area includes the initialization parameter settings of the PSO algorithm, such as the number of particles, the number of particle iterations, and the fitness value. These settings include all the values that the problem application needs to initialize. The application can receive the settings from the parameter area according to its own data conditions and needs. The evaluated data is compared in Figure 4.

The solution is represented by “PS0 1” in the system, and the PSO algorithm based on self-balancing is represented by “PSO” in the system. Z” means that the self-balancing PSO algorithm of parallel processing is represented by “M PSO 2” or “MO PSO 2” in the system, which uses a progressive method to reflect the algorithm's solving ability and speed in line with people's perception of things. *Way of Thinking*. In order to make the solution result of the TSP problem clearer and not be disturbed by the urban road network data, the solution result in the TSP problem area will be output by displaying the path trajectory and path length in the text box. According to the aforementioned application model of the PSO algorithm in the TSP problem, the overall flow chart of the TSP problem model is shown in Figure 5.

In the above model flow chart, the key issue is to regularize the data according to the specific map data and design an algorithm that can solve the problem. By using the geographic coordinates in the data to calculate the distance between tourist attractions using formulas, it is ensured that the particle swarm algorithm can solve this TSP problem. According to the number of different particles and the number of iterations, the particle swarm algorithm can find the optimal path or better path under the control of the self-balancing mechanism. The parallel processing of the algorithm will also be a breakthrough in the specific application of the parallel model. Each algorithm in the design will solve the TSP problem according to the value provided in the parameter area and output the final result to the system interface.

In the above-mentioned areas, no matter which area is in the system, they follow the following steps:

(l) Load map data and adjust display map data
(2) Enter the required parameters in the parameter area
(3) Click the corresponding algorithm to solve the problem
(4) Display the path trajectory and output the path length

## 4. Experimental Research

In order to show the research results, this article uses the ArcGIS Engine platform and ArcGIS Engine to develop a desktop application of a travel route planning system based on the Viterbi algorithm, which allows users to choose the starting point of travel, the number of travel days, and the type of travel, and then automatically calculate the most suitable for requirements.

*Travel Path*. After calculating the parameters, the data needs to be processed. First, import the data into ArcMap, and assign attribute values to each scenic spot and hotel, among which the data of user evaluation level and consumption level come from the Internet. The maximum longitude of all scenic spots and hotels in this article is 114.42°, the minimum value is 114.21°, the maximum latitude is 30.68°, and the minimum is 30°. 50°, NR˜20 is obtained from all the above data. 006, NC˜19.998. Then, open the Fishnet function in ArcMap and input the above data to generate a 20 × 20 grid. Finally, overlay the generated grid with scenic spots and hotels to generate Intersect_Fishnet_Sceinc and Intersect_Fishnet_Hotel layers. At this time, the grid coordinates, grades, names, and user reviews of scenic spots and hotels can be obtained in the attribute table of the new layer. All information has a consumption level. The predicted value is shown in Figure 6.

This article assumes four different scenarios. As shown in Table 1, the conditions of each scenario are different from each other, corresponding to the needs of different tourists.

In Experiment 1, the tourists chose “Wuhan University” as the starting point. The next attraction of “Wuhan University” is the “Hubei Provincial Museum”, which has free tickets and a wealth of collections. The visit value is extremely high, and it is one of the most cost-effective scenic spots in Wuhan. It is about 4 km away from “Wuhan University” and the distance is moderate. The hotel searched for is “Hanting Hotel (Donghu Branch)”, which has a high score on travel websites such as “Ctrip”. The hotel has an excellent location, close to Metro Line 4, affordable, and only a short distance from “Hubei Provincial Museum”. 1 km, so the planned route as a whole meets user requirements. The algorithm convergence diagram is shown in Figure 7.

Experiments 2, 3, and 4 are all comparative experiments of Experiment 1. In Experiment 2, only the travel type was changed, and the next scenic spot retrieved became “Chu River Han Street”. This scenic spot belongs to the shopping and entertainment type and is surrounded by 3 large commercial districts. Therefore, the per capita consumption is relatively high. 5 km, within a moderate distance, the searched hotel is a five-star hotel in Wuhan, which is about 0.5 km away from “Chu River Han Street”. 2 km, the planning result is very in line with the requirements of comfortable tourism. In Experiment 3, the travel time was changed, and it was found that the travel path of Experiment 1 was the same as that of Experiment 3 on the first day. It can be seen that the characteristics of the Viterbi algorithm from the local optimal to the overall optimal; Experiment 3, the second day of “East Lake Ocean World.” As a starting point to start the search, there are many attractions within 15 km of the attraction, but the only relatively close ones are “Chu River Han Street” and “Wuhan Happy Valley”. These two attractions have a greater impact on the planning results. Although the distance from “Wuhan Happy Valley” to the starting point is closer, due to the existence of consumption levels, the final calculation result is that “Chu River Han Street” is better than “Wuhan Happy Valley”. Observation state probability and state transition probability affect each other. Finally, in Experiment 4, only the starting point was changed, but from the calculation results, there is no essential difference from Experiment 1.

From the above experiments, it can be concluded that the travel route planning based on the Viterbi algorithm makes full use of the dynamic planning method of the Viterbi algorithm, which not only considers the distance between tourists and scenic spots and hotels but also combines the tourists' own travel needs. The quoted Gaussian function can better express the relationship between distance and state transition probability; the setting of tourism type allows tourists to diversify their choices. The optimal path is shown in Figure 8. The predicted value is compared in Figure 9, which can be seen the optimized one is better.

## 5. Conclusion

This article explores the particle swarm model in tourism path planning and innovatively proposes to add hotels to tourism path planning, which increases the practicality of tourism path planning and uses grids to express the spatial location relationship of scenic spots and hotels, use Gaussian function to express the probability of observation state, and use the attributes of scenic spots and hotels to express the probability of state transition; finally, the Viterbi algorithm is successfully combined with the above methods to realize the Viterbi tourism path planning algorithm, and the results are verified by experiments. It shows that the algorithm is reasonable and meets the multifactor path planning needs of users to a certain extent. However, this algorithm also has its shortcomings. For example, replacing the actual distance with the Manhattan distance under the grid model will inevitably produce errors. In future research, other clustering methods can be explored to minimize errors. The planning result is more accurate.

Nowadays, China's information industry is developing rapidly. The combination of tourism and GIS has gradually improved the information level, but there is still a lot of room for development. In future applications, a national optimal travel route website or travel route query decision-making system can be established, and travel route planning can be extended to specific road planning. The level of development and perfection of tourism routes play a role in controlling the flow and direction of tourism; at the same time, it can alleviate the congestion during peak tourism period, can effectively improve the overall tourism quality of tourists, and is of great significance to the development of China's tourism industry.

However, in mature research, most of the research environment is carried out in a static environment, that is, the obstacle is fixed, but the situation that the obstacle changes with time is still lacking. This is also should be done in the future.

## Figures and Tables

**Figure 1:** Tourism route design.

**Figure 2:** Global optimal solution.

**Figure 3:** Predicted value.

**Figure 4:** Evaluated data.

**Figure 5:** TSP problem model.

**Figure 6:** Prediction.

**Figure 7:** Algorithm convergence diagram.

**Figure 8:** Optimal path.

**Figure 9:** Comparison of value.

**Table 1:** Experiment details.

Item	Starting point	Time/d	Type
Experiment 1	Wuhan University	1	Economical
Experiment 2	Wuhan University	1	Economical
Experiment 3	Wuhan University	2	Economical
Experiment 4	Jianghan road	1	Economical

## Data Availability

The data used to support the findings of this study are available from the corresponding author upon request.
